# Regenerative Medicine for the Cornea

**DOI:** 10.1155/2013/428247

**Published:** 2013-12-17

**Authors:** Yoshinori Oie, Kohji Nishida

**Affiliations:** Department of Ophthalmology, Osaka University Graduate School of Medicine, 2-2 Yamadaoka, Suita, Osaka 565-0871, Japan

## Abstract

Regenerative medicine for the cornea provides a novel treatment strategy for patients with corneal diseases instead of conventional keratoplasty. Limbal transplantation has been performed in patients with a limbal stem cell deficiency. This procedure requires long-term immunosuppression that involves high risks of serious eye and systemic complications, including infection, glaucoma, and liver dysfunction. To solve these problems, ocular surface reconstruction using cultured limbal or oral mucosal epithelial stem cells has been successfully applied to patients. However, cell sheets must be fabricated in a cell processing center (CPC) under good manufacturing practice conditions for clinical use, and the expenses of maintaining a CPC are too high for all hospitals to cover. Therefore, several hospitals should share one CPC to standardize and spread the application of regenerative therapy using tissue-engineered oral mucosal epithelial cell sheets. Consequently, we developed a cell transportation technique for clinical trial to bridge hospitals. This paper reviews the current status of regenerative medicine for the cornea.

## 1. The Structure of the Cornea

The cornea is an avascular and transparent tissue that forms part of the anterior ocular segment. Together with the sclera, it forms the outer shell of the eyeball. The cornea serves as the transparent window of the eye that allows light to enter, whereas the sclera provides a dark box that allows an image to form on the retina. The cornea is exposed to the outer environment, whereas the white sclera is covered with the semitransparent conjunctiva and is not directly exposed to the outside.

The central cornea is 515 *μ*m thick [1]. It comprises an outer stratified squamous nonkeratinized epithelium, an inner connective tissue stroma, and the innermost layer, a cuboidal endothelium (Figure 1). Disorders in any of these layers can cause corneal opacity and visual disturbance: epithelial disorder (e.g., limbal stem cell deficiency), stromal disorder (e.g., corneal dystrophy), and endothelial disorder (e.g., bullous keratopathy).

## 2. Limbal Stem Cells

The corneal epithelium has five to seven cell layers and is 50–52 *μ*m thick. It is composed of small basal cells, flattened middle cells (wing cells), and polygonal flattened superficial cells. Corneal epithelial stem cells (limbal stem cells) are thought to reside in the basal layer of the limbus, the transitional zone between the cornea and the conjunctiva (Figure 2) [2, 3]. Transient amplifying (TA) cells are generated by stem cells and then migrate into the central cornea. Although stem cells are low-cycling, TA cells proliferate rapidly.

Thoft and Friend hypothesized that corneal epithelial maintenance can be defined by the equation *X* + *Y* = *Z*, with *X* being the proliferation of basal epithelial cells; *Y* being the contribution to the cell mass by the centripetal movement of peripheral cells; and *Z* being the epithelial cell loss from the surface [4]. Therefore, the proliferation and migration of TA cells differentiated from stem cells play very important roles in the maintenance of corneal epithelium.

p63, ATP-binding cassette subfamily G member 2 (ABCG2), N-cadherin, K19, NGF receptors (TrkA), and integrin a6 have been reported as candidate markers of limbal stem cells. However, a specific marker has not yet been identified [4–9].

The palisades of Vogt are distinctive normal features of the human corneoscleral limbus [10] (Figure 3). They are more discrete in younger and more heavily pigmented individuals, and they appear more regular and prominent at the lower limbus than at the upper limbus. They are observed infrequently along the horizontal meridian.

Lately, a new phenomenon, “limbal epithelial crypts (LEC),” has been reported as a putative limbal stem cell niche [11, 12]. Cells within LEC have the phenotype of CK3−/CK19+/CD34−/Vimentin+/p63+/Connexin43+/MlB (Ki67)−.

## 3. Limbal Stem Cell Deficiency

If limbal stem cells are completely absent, vascularized conjunctival epithelium invades into the cornea. The condition is called limbal stem cell deficiency (LSCD) (Figure 4). It results in a corneal neovascularization and opacification that disturbs visual acuity. The causative diseases can be classified into four groups: (1) congenital diseases caused by congenital aplasia of stem cells (e.g., aniridia, sclerocornea); (2) diseases with an external cause, involving the loss of stem cells due to trauma (e.g., thermal, alkali, and acid burns); (3) diseases involving internal, stem cell exhaustion, such as Stevens-Johnson syndrome and ocular cicatricial pemphigoid; and (4) idiopathic diseases of unknown cause [13].

## 4. Limbal Transplantation

In patients with unilateral limbal stem cell deficiency, autologous limbal transplantation can be used to achieve surface reconstruction of the cornea [14]. However, this procedure requires a large limbal graft from the healthy eye (incurring a risk of causing limbal stem cell deficiency in the healthy eye [15]) and is not applicable to bilaterally affected patients [16]. Limbal-allograft transplantation can be performed in patients with unilateral or bilateral deficiencies [17, 18]. However, it has two main problems: postoperative complications and a donor shortage.

Postoperative complications include rejection and bacterial or fungal keratitis [19–22]. Limbal transplantation requires long-term immunosuppression, which involves high risks of serious eye and systemic complications, including infection and liver and kidney dysfunction. Even with immunosuppression, graft failure is common in patients with Stevens-Johnson syndrome or ocular pemphigoid due to serious preoperative conditions, such as persistent inflammation of the ocular surface, abnormal epithelial differentiation of the ocular surface, severe dry eye, and lid-related abnormalities.

Donor shortage is also a major problem in many countries, including Japan. The Japan Eye Bank Association reported that the number of patients waiting for keratoplasty was 2,286 but that the number of donors was 891 in Japan in 2012.

## 5. Regenerative Medicine and Tissue Engineering

Langer and Vacanti established the field of “tissue engineering” [23, 24]. Tissue engineering is an interdisciplinary field that applies the principles of engineering and the life sciences toward the development of biological substitutes that restore, maintain, or improve tissue function. This technology has been applied to various tissues and organs, including the skin, cornea, cartilage, and heart [25–34]. Enormous promise has been ascribed to this technology because it offers a paradigm shift from conventional organ transplantation to a novel treatment strategy that relies on cultured stem cells. Furthermore, this technique could potentially solve the two main problems of corneal transplantation.

## 6. Cultivated Limbal Epithelial Cell Transplantation (CLET)

Autologous cultivated limbal epithelial cell transplantation was initially reported by Pellegrini and colleagues [26]. They reported that two patients with LSCD caused by alkali burns were restored using autologous cultivated corneal epithelium, and the outcome persisted for more than two years after grafting. This report is the first of a clinical application in the field of regenerative medicine for the cornea.

Following this report, many investigators have reported the effectiveness and safety of CLET [35–39]. The amniotic membrane and fibrin glue have been mainly used as substrates for cultivated cells. The amniotic membrane has been used as a natural substrate because it can expand into the stem cell niche [40]. Various cytokines released from the amniotic membrane, such as epidermal growth factor, keratinocyte growth factor, hepatocyte growth factor, nerve growth factor, and basic fibroblast growth factor, have been reported to play important roles within the niche of limbal stem cells. The amniotic basement membrane offers a basement membrane for corneal epithelial cell adhesion.

Rama et al. recently reported long-term corneal regeneration using autologous cultivated limbal stem cells [29]. They showed that permanent restoration and a renewal of the corneal epithelium were achieved in 76.6% of 107 eyes with LSCD caused by chemical and thermal burns, and the success of the ocular surface reconstruction was significantly associated with the percentage of p63-bright, holoclone-forming stem cells in culture. No severe adverse events were observed. Their results demonstrated the effectiveness and safety of CLET and the importance of the stem cell population within the cultured cells.

## 7. Cultivated Oral Mucosal Epithelial Cell Transplantation (COMET)

Although CLET can be applied to patients with unilateral LSCD, it cannot be applied to patients with bilateral disease because they have completely lost their own limbal stem cells as a cell source. Consequently, autologous cultivated oral mucosal epithelial cell transplantation (COMET) has been developed for patients with bilateral LSCD [28, 41]. Even in unilateral cases, some patients wish to avoid tampering with the limbus of their unaffected eye.

We use a temperature-responsive culture dish to fabricate oral mucosal cells [42]. Cell sheets are cultivated on the dishes coated with a temperature-responsive polymer, poly(N-isopropylacrylamide) (PIPAAm), which is hydrophobic below 32°C and hydrophilic above 32°C (Figure 5). This change releases the cell sheet, allowing it to be removed without destroying the cell-cell or the cell-extracellular matrix interactions within the cell sheet. Therefore, cultivated oral mucosal epithelial cells can be harvested using a temperature reduction without the use of enzymes.

The cell morphology of an oral mucosal epithelial cell sheet fabricated on a temperature-responsive culture dish is similar to that of the normal cornea or a corneal epithelial cell sheet (Figure 6). It consists of approximately four epithelial layers, flattened superficial cells, and small basal cells with a high C/D ratio. Keratin 3/76, a marker of corneal and oral mucosal epithelium, is positive in the oral mucosal epithelial cell sheet. p63, a putative stem cell marker, is positive for basal cells. ZO-1, a marker of tight junctions, is positive, particularly between superficial cells. The oral mucosal epithelial cell sheet is assumed to have a similar phenotype to that of corneal epithelium as well as enough stem cells and a barrier capability for ocular surface reconstruction. We have already begun a clinical study using this technique and achieved favorable results (Figure 7) [28].

There has been no report on severe adverse events including development of malignant tumor following COMET. However, if there is a problem, we can easily observe and remove transplanted oral mucosal cells from ocular surface. From that point of view, ocular surface would be the ideal environment for application of this kind of new treatment.

Longstanding survival of transplanted oral mucosal epithelial cells remains unclear. Because autologous oral mucosal cells are used as a cell source, there is no method to distinguish transplanted cells and native cells from host tissue. Even if phenotype of transplanted oral mucosal epithelial cells is maintained, there remains the possibility that host conjunctival cells invaded into cornea and changed the phenotype. However, analyses on phenotype of corneal epithelium excised during keratoplasty following COMET suggest longstanding survival of transplanted oral mucosal epithelial cells. Nakamura et al. reported that phenotype of transplanted cultivated oral epithelial cells (keratin 3[+], Muc5ac[−]) was maintained in clinically successful COMET grafts, and the phenotype was not maintained in failed grafts [43]. Chen et al. showed that all specimens were unanimously positive for K3, -4, and -13 but negative for K8 and MUC5AC, suggesting that the keratinocytes were oral-mucosa-derived [44].

Ohki et al. also applied tissue-engineered oral mucosal epithelial cell sheets to prevent esophageal stricture after endoscopic submucosal dissection [45]. Oral mucosal epithelial cells can be applied for other diseases in the future.

## 8. Transportation Technique for Regenerative Medicine

The cell sheets must be fabricated in a cell processing center (CPC) under good manufacturing practice (GMP) conditions for clinical use. However, the expenses for a CPC are extremely high, and it is impossible for all hospitals to cover the cost. Therefore, multiple hospitals should share one CPC to standardize and spread regenerative therapy using tissue-engineered oral mucosal epithelial cell sheets. Therefore, the development of cell transportation techniques is necessary for bridging many hospitals.

We developed a transportation container with three basic functions: maintaining a constant interior temperature, air pressure, and sterility (Figure 8) [46]. The interior temperature and air pressure were monitored by a sensor. Human oral mucosal epithelial cells obtained from two healthy volunteers were cultured on temperature-responsive culture dishes. The epithelial cell sheets were transported via airplane between Osaka University and Tohoku University using the developed cell transportation container. Histological and immunohistochemical analyses and flow cytometric analyses for cell viability and cell purity were performed on the cell sheets before and 12 h after transportation to determine the effect of transportation on the cell sheets. Sterility tests and screening for endotoxins and mycoplasma in the cell sheets were performed before and after transportation.

During transportation via airplane, the temperature inside the container was maintained above 32°C, and the air pressure did not fluctuate more than 10 hPa. The cell sheets were well stratified and successfully harvested before and after transportation (Figure 9). The expression patterns of keratin 3/76, p63, ZO-1, and MUC16 remained consistent before and after transportation. The cell viability was 72.0% before transportation and 77.3% after transportation. The epithelial purity was 94.6% before transportation and 87.9% after transportation. Sterility tests and screening for endotoxins and mycoplasma were negative for all cell sheets.

We are conducting a multicenter clinical study using the transportation technique described herein (Figure 10). In this clinical study, we will harvest oral mucosal epithelial tissues from patients at institute 1 and transport them to institute 2. At institute 2, a cell sheet will be fabricated at the CPC. Next, the cell sheet will be sent to institute 1 for transplantation. We will culture oral mucosal epithelial cells from two other institutes in Osaka University. Culturing at a single CPC enables better control of the quality of the tissue-engineered human oral mucosal epithelial cell sheet. If this effort is successful, we will be able to treat many patients in many hospitals all over the world without the need for a CPC.

The newly developed transportation technique for air travel is an essential technology for regenerative medicine and promotes the standardization and spread of regenerative therapies.

## 9. Conclusion

Many researchers have engaged in basic and clinical study in the fields of stem cell and regenerative medicine for the cornea. However, there are no government-approved tissue-engineered medical products for the cornea so far. Although first-in human clinical study using a novel cell source or technology is both sensational and impressive, efforts to turn this established technique into a standardized therapy should be a continuous process. We are struggling to make oral mucosal epithelial cell sheets an approved medical device. We believe that, once approved, this medical product will help visually impaired patients all over the world and that this goal can be achieved in the near future.

## Figures and Tables

**Figure 1:** The structure and disorders of the cornea. The cornea consists of three layers: epithelium, stroma, and endothelium. Visual acuity can be affected by disorders of any of these layers, including limbal stem cell deficiency, corneal dystrophy, and bullous keratopathy.

**Figure 2:** Limbal stem cells. Limbal stem cells are believed to be located within the basal layer of the limbus. Transient amplifying (TA) cells are progenitor cells that differentiate from limbal stem cells and then migrate into the central cornea.

**Figure 3:** Palisades of Vogt (POV). A slit lamp examination reveals the limbus-specific feature, the “palisades of Vogt” (POV).

**Figure 4:** Slit lamp photographs of patients with a limbal stem cell deficiency. (a) Aniridia; (b) alkali burn; (c) ocular cicatricial pemphigoid; (d): Stevens-Johnson syndrome.

**Figure 5:** Ocular surface reconstruction via the autologous transplantation of tissue-engineered cell sheets fabricated from oral mucosal epithelial cells. Oral mucosal tissue containing whole epithelial cell layers was excised from the oral cavities of the patient. The cells were then seeded onto a temperature-responsive culture dish. The cultured cells were harvested as a cell sheet by reducing the culture temperature. The cells were then transplanted onto the corneal surfaces of the patient.

**Figure 6:** Histological and immunohistochemical analyses of cell sheets. HE staining was performed for an oral mucosal epithelial cell sheet (a), a normal cornea (b), and a corneal epithelial cell sheet (c). Human oral mucosal epithelial cell sheets were stained with antikeratin 3/76 (d), anti-p63 (e), and anti-ZO-1 (f) antibodies. Nuclei were costained with Hoechst 33342. Scale bars: 50 *μ*m.

**Figure 7:** Slit lamp photographs of patients before and after cultivated oral mucosal epithelial cell transplantation. (a) The right eye has a total limbal stem cell deficiency caused by ocular cicatricial pemphigoid. The VA is 20/2000. (b) Eight years postoperatively, the corneal epithelial clarity was well maintained. The VA is 20/222 despite macular degeneration.

**Figure 8:** Cross-sectional view of a cell transportation container for cell sheets, consisting of an incubation vessel for temperature, a sealing apparatus for air pressure, and four packaging chambers for sterility. Bottles with heat storage material are set inside the incubation vessel.

**Figure 9:** Human oral mucosal epithelial cell sheets before and 12 h after transportation. The cell morphology was examined using phase-contrast microscopy (a, b) and HE staining (c, d). Scale bars: 100 *μ*m (a, b), 50 *μ*m (c, d).

**Figure 10:** Multicenter clinical study of a cell sheet transportation system. Oral surgery for mucosal tissue and cell sheet transplantation are performed at institute 1; the cell sheets are cultured in the CPC at institute 2.
